This article has been retracted.

# The impact of Fosetyl-Aluminium application timing on Karnal bunt suppression and economic returns of bread wheat (*Triticum aestivum* L.)

**DOI:** 10.1371/journal.pone.0244931

**Published:** 2021-01-11

**Authors:** Muhammad Arif, Sagheer Atta, Muhammad Amjad Bashir, Muhammad Ifnan Khan, Ansar Hussain, Muhammad Shahjahan, Mona S. Alwahibi, Mohamed Soliman Elshikh

**Affiliations:** 1 Department of Plant Protection, Faculty of Agricultural Sciences, Ghazi University, Dera Ghazi Khan, Pakistan; 2 Department of Plant Breeding and Genetics, Faculty of Agricultural sciences, Ghazi University, Dera Ghazi Khan, Pakistan; 3 Department of Plant Pathology, Faculty of Crop and Food Sciences, PMAS, Arid Agriculture University, Rawalpindi, Pakistan; 4 Department of Botany and Microbiology, College of Science, King Saud University, Riyadh, Saudi Arabia; Harran University, TURKEY

## Abstract

Fungal pathogens exert severe qualitative and quantitative damages to wheat crop. Karnal bunt of wheat caused by *Tilletia indica* Mitra, Mundkur is a severe threat to global food security. Nonetheless, *T*. *indica* is regulated as a quarantine pest in numerous countries, which further aggravates the situation. Tolerant varieties and appropriate management practices for Karnal bunt are imperative to meet the global wheat demands. This two-year study explored the impact of fungicide [Fosetyl-Aluminium (Aliette)] application timing on allometric traits, disease suppression and economic returns of bread wheat. Four bread wheat cultivars differing in their tolerance to Karnal bunt were used in the study. Fungicide was applied as either seed treatment (ST), foliar application at heading (FAH) or ST + FAH, whereas no application (NA) was taken as control. Lasani-08 performed better than the rest of the cultivars in terms of allometric traits (plant height, leaf area, crop growth rate, photosynthesis, and chlorophyll content), yield and economic returns. Nonetheless, minimal disease severity was recorded for Lasani-08 compared to other cultivars during both years. The ST improved allometric traits of all cultivars; however, ST + FAH resulted in higher yield and economic returns. Cultivar Pasban-90 observed the highest disease severity and performed poor for allometric traits, yield and economic returns. It is concluded that ST + FAH of Fosetyl-Aluminium could be a pragmatic option to cope Karnal bunt of wheat. Nonetheless, Pasban-90 must not be used for cultivation to avoid yield and quality losses.

## Introduction

Bread wheat (*Triticum aestivum* L.), a member of Poaceae is staple food for one third of the global population. It contributes ~21% towards global energy needs. It provides income for farmers in many countries of the world. Globally, wheat is cultivated on ~21.42 million hectares with 734 million tons annual production [1, 2]. Global average wheat yield is far below than its yield potential. Numerous biotic and abiotic factors are responsible for this low productivity. Biotic factors include many important pathogens like fungi, nematodes, viruses and bacteria. Fungi have become main disease-causing agents in wheat. The diseases caused by fungi include rust, smut and bunt. These diseases cause severe qualitative and quantitative losses in wheat every year [3, 4].

Karnal bunt (KB) of wheat was firstly identified in 1931 from Indian town Karnal; thus, named as Karnal bunt [5]. The KB spread rapidly to different regions of India and neighboring countries, including Pakistan, Afghanistan, Nepal, Iran, Iraq, Mexico and partially in areas of Australia, the United States, Brazil and South Africa [6, 7]. The KB is caused by air, soil-seed borne fungal pathogen *Tilletia indica* Mitra, Mundkur, which is categorized by auxiliary part of seed having black powdery growth [6].

The disease mostly appears in wheat growing areas with low winter temperature and high relative humidity. The KB appeared in many countries after wheat imports [8]. International transportation of agricultural commodities, globalization, trade liberalization and climate change have enhanced the chances of KB spread. Host-pathogen interface has also become a main factor for disease incursion. Different resistant foundations for KB have been already recognized and applied for breeding of resistance resource. Newly identified high standard genomes of mono-teliospores culture of KB are working as an encouraging mean for understanding the pathogenicity and development of the fungus [9].

The KB directly affects grain quality and weight through production of foul, fleshy smell [10]. Breeding programs to confer the resistance against KB are fundamental approaches and optimal methods to cope with the disease. Wheat is vulnerable to KB due to which Food and Agriculture Organization (FAO) and International Maize and Wheat Improvement Center (CIMMYT) send fresh lines/cultivars to different countries for checking their resistance against the disease under different ecological zones [6]. Classification and identification of resistant genes is most important tactic for identifying molecular mechanisms of disease tolerance [7, 11].

The dispersal of *T*. *indica* teliospores occurs naturally. Germinating teliospores can discharge abundant spores in soil, which produce sporicidal masses for infection on wheat florets. Application of different fungicides, including Agrozim fentin hydroxide, Bavistin (Carbendazim), Propioconazole, Biteranol and Bayleton (Triadimefon) during flowering or late booting stage can minimize the disease incidence. Application of propioconazole during the anthesis has significantly suppressed *T*. *indica* [9, 12].

*T*. *indica* is seed inhabited, airborne, can profound in soil and have penetrative ability to host plants under favorable conditions. Application of antifungal agents like seed dressing with fungicides and biocontrol agents are effective management strategies. Environmental dynamics play a significant role in the development of KB. Wheat crop is susceptible to KB at different developmental stages [13]. Some studies have revealed the conceived generic placement and evolutionary relationship of KB species with other pathogens [14].

With the exclusion of some mercurial fungicides forbidden in many countries, seed treatments with fungicides have become unsuccessful in managing teliospores of KB. One major aftermath of seed treatment is the antagonistic effect on seed germination of wheat. Nonetheless, inoculum of *T*. *indica* can be minimized by applying guanidine fungicides, cyano (methylmercuric) and hexacholorobezene as seed treatment. Several other fungicidal products are also efficient in managing teliospores [1, 15]. Chemical management of KB is possible with the help of triazole fungicides during heading period [16]. Several fungicides applied against KB teliospores work as fungistatic. Resistant source in term of disease-free seed can be obtained by applying the propioconazole 0.1% on heading stage [17]. Recent studies regarding the management of KB with the help of fungicides revealed that propioconazole has become a significant fungicide in managing the disease by chemical control.

However, the impact of fungicide application on disease suppression, allometry and economic returns of wheat cultivars with varying inherent tolerance to KB have merely been tested. The current study inferred the impact of fungicide application timing on allometry, disease severity index and economic returns of four wheat cultivars differing in their tolerance to KB.

## Materials and methods

### Experimental site

This two-year study was conducted at farmers’ field at Alipur (29.382263°N, 70.920865°E). The study did not require any permit and involved no endangered species. The area lies in semi-arid region, with high summer temperature and moderate winters. Soil of the experimental site was clay-loam. Soil samples were collected and analyzed prior to experiments. Climatic data regarding temperature, relative humidity and sunshine hours were collected with Hobo data logger. Rainfall data were collected from the nearest meteorological station. The soil properties of the experimental site and climatic data of both years are summarized in Tables 1 and 2, respectively.

**Table 1:** Physiochemical characteristics of experimental soil before initiation of the experiment during both the years of study.

Soil properties	Unit	Years		Soil properties	Unit	Years	
		2016–17	2017–18			2016–17	2017–18
Chemical Analysis				Physical analysis			
Organic matter content	%	0.54	0.49	Silt	%	53.10	50.20
Total nitrogen (N)	%	0.14	0.16	Sand	%	24.10	28.10
Available phosphorus (P)	mg kg^-1^	7.21	8.01	Clay	%	23.80	22.70
Available potassium (K)	mg kg^-1^	222.19	219.23	Textural class		Silty-clay	Silty-clay
pH		8.02	8.23				
EC	dS m^-1^	2.91	2.68				

**Table 2:** Weather data of experimental site during both years of the study.

Month	T (°C)	RH (%)	Sunshine	Rainfall	T (°C)	RH (%)	Sunshine	Rainfall
			(hours)	(mm)			(hours)	(mm)
2016–17					2017–18			
November	18.8	71.6	3.2	0.0	18.2	80.6	3.4	6.2
December	15.2	77.4	3.1	0.0	15.5	76.8	4.2	14.0
January	11.9	81.8	3.2	12.7	12.8	82.9	5.4	0.0
February	15.3	79.8	6.3	13.0	16.7	76.5	5.9	5.6
March	20.8	71.4	6.2	2.1	22.9	73.2	7.8	22.0
April	31.2	56.5	6.1	7.8	30.8	60.7	7.2	10.0

T = average temperature, RH = relative humidity, the values are monthly averages

### Experimental details

The experiment consisted of two factors, i.e., wheat cultivars and fungicide application timing. Four wheat cultivars differing in their susceptibility to *Tilletia indica* were included in the study (Table 3). Seeds of the cultivars were procured from Regional Agricultural Research Institute, Bahawalpur. Seeds were surface sterilized with sodium hypochlorite. The experiments were conducted during rabi cropping seasons of 2017–18 and 2018–19. Fosetyl-Aluminium (Aliette® WG 80WP) systemic fungicide was used for seed treatment (ST) and foliar application at heading (FAH). Fostyl-Aluminium belongs to organophosphorus group having chemical formula [C_2_H_5_OP(H)O_2_]_3_Al and derived from ethylphosphate [18]. Same concentration (250g/100 liter of water) of fungicide was applied on all cultivars as ST, FAH and ST + FAH. The fungicide was applied as ST, FAH or ST + FAH, while no application (NA) was regarded as control treatment. Seeds were sown on November 21 and 23 during 2017–18 and 2018–19, respectively. A 1-meter canola buffer zone was created between the plots to exclude the damage of airborne spore dispersal. Seeds were sown with a manual drill keeping row-to-row distance of 20 cm. The net plot size was 4 × 10 m, while each treatment had four replications.

**Table 3:** Different wheat cultivars used in the study with their tolerance/susceptibility level to Karnal bunt of wheat.

Cultivar	Susceptibility
Lasani-08	Moderately resistant *(1R)*
Faisalabad-08	Moderately susceptible (*1S)*
Abdul Sattar-2002 (AS-02)	Susceptible *(2S)*
Pasban-90	Highly susceptible *(3S)*

### Data collection

Data relating to allometric traits, yield-related parameters and disease severity index were recorded using standard procedures.

### Allometric traits

Leaf area was recorded by destructive method. Leaf area was recorded at biweekly intervals from 35 days after sowing (DAS) using a leaf area meter (DT Area Meter, model MK2; Delta-T Devices, Cambridge, UK). A 0.5 m^2^ area was cut, weighed and area of pre-weighed leaves was measured. Leaf area index (LAI) was calculated as the ratio of leaf area to ground area [19]. Leaf growth rate (LGR), crop growth rate (CGR) and net assimilation rate (NAR) were computed according to the procedures devised by Hunt [20, 21].

### Yield-related parameters

The crop was harvested at maturity to record yield-related attributes. Total number of grains on ten randomly selected spikes were counted and averaged for recording number of grains per spike. Three random samples of 1000 grains from each experimental unit were weighed and averaged to get 1000-grain weight. Each experimental unit was harvested manually, tied into bundles and sundried for one week. These bundles were threshed manually, grains were separated and weighed to record grain yield. The yield was converted to kg ha^-1^ by unitary method.

### Disease severity index

For comparison of different cultivars in terms of resistance to KB, disease severity index was calculated [22, 23]. Resistance and susceptibility levels of the cultivars were calculated by a disease rating scale [24]. Disease severity index was calculated by formula given below;

$$\text{Disease}\;\text{severity}\;\text{index}(\%)=\frac{\sum (\text{Class}\;\text{frequency}\times \text{rating}\;\text{class}\;\text{score})}{\text{Total}\;\text{number}\;\text{of}\;\text{observations}}\times 100$$

### Statistical analysis

The collected data were tested for normality and homogeneity of variance first, which indicated normal distribution. Paired *t* test was used to infer the differences among years, which indicated significant differences. Therefore, data of both years were analyzed and presented separately. Two-way analysis of variance (ANOVA) was used to infer significance in the data [25]. Least significant difference test at 95% probability level was used as a post-hoc test to separate the means. Allometric traits were presented in the form of line graphs using means ± standard errors of means. All statistical analyses were performed on SPSS version 20.0 [26] and graphs were created in Microsoft Excel version 2016.

### Economic analysis

The economics of fungicide application on different wheat cultivars was computed by economic analysis. Costs incurred on seed procurement, land preparation, seed sowing, weed management, irrigation, fertilizer application, harvesting, fungicide and its application, land rent for six months and labor cost were added to compute total expenses incurred. Existing market price for wheat grain and straw were used to compute gross income. Net income was calculated by subtracting the total expenses from gross income and the benefit-cost ratio (BCR) was calculated by dividing gross income by the total cost of production.

## Results and discussion

### Allometric traits

Different allometric traits, i.e., leaf area index (LAI), leaf growth rate (LGR), crop growth rate (CGR), net assimilation rate (NAR), photosynthesis and chlorophyll contents were recorded during both years. Allometric traits improved with time, reached to the highest level and then started to decline (Figs 1–4). The studied allometric traits differed among wheat cultivars included in the study. Better allometric traits were recorded for Lasani-08, whereas Pasban-90 resulted in poor allometric traits during both years. Fungicide application at different growth stages altered allometric traits and the highest improvement was recorded for ST compared to NA during each year (Figs 1–4).

**Fig 1:** The influence of different fungicide application timings on leaf area index of wheat cultivars with varying tolerance to Karnal bunt disease.

**Fig 2:** The influence of different fungicide application timings on leaf growth rate of wheat cultivars with varying tolerance to Karnal bunt disease.

**Fig 3:** The influence of different fungicide application timings on crop growth rate of wheat cultivars with varying tolerance to Karnal bunt disease.

**Fig 4:** The influence of different fungicide application timings on net assimilation rate of wheat cultivars with varying tolerance to Karnal bunt disease.

Studies on plant pathogen connections are continually flourishing because of development novel methods and computational powers. Various aspects of plant pathogens interactions with respect to climate change and agricultural practices have necessitated the development of durable pest/pathogen resistance in many agricultural crops [27]. Better allometric traits with ST can be owed to lowered teliospores germination compared to NA. Nonetheless, allometric traits reach to their highest value until heading stage. Therefore, FAH could not contribute much towards allometric traits.

Wheat cultivars, fungicide application timing and their interaction significantly altered plant height, chlorophyll contents and photosynthesis during both years. The highest plant height, chlorophyll contents and photosynthesis were recorded for Lasani-08, whereas Pasban-90 had the lowest values of these traits during each year. Similarly, ST observed the highest values of plant height, while NA had the lowest values of these parameters during both years (Table 4). Nonetheless, ST + FAH had the highest chlorophyll contents and photosynthesis during both years, whereas NA observed the lowest values of these parameters. Regarding cultivars × fungicide application timings’ interaction, Lasani-08 with ST + FAH had the highest plant height, chlorophyll contents and photosynthesis, whereas Pasban-90 with NA recorded the lowest plant height, chlorophyll contents and photosynthesis during both years (Table 4).

**Table 4:** The impact of fungicide application timing on allometric traits and disease severity index of different wheat cultivars with varying tolerance to Karnal bunt disease.

	2016–17				2017–18			
	Plant height	Photosynthesis	Chlorophyll	DSI	Plant height	Photosynthesis	Chlorophyll	DSI
**Varieties (V)**								
**V**_**1**_	101.42 a	15.09 a	2.75 a	2.04 d	102.98 a	14.12 a	2.48 a	2.18 d
**V**_**2**_	94.42 b	13.51 b	2.48 b	2.71 c	96.88 b	12.48 b	2.19 b	2.84 c
**V**_**3**_	89.00 c	12.02 c	2.28 c	2.94 b	91.58 c	10.74 c	2.04 c	3.26 b
**V**_**4**_	77.42 d	11.23 d	1.88 d	3.94 a	80.10 d	10.08 d	1.62 d	4.02 a
**LSD**	**1.59**	**0.32**	**0.08**	**0.03**	**1.59**	**0.32**	**0.08**	**0.04**
**Application Timing (T)**								
**T**_**1**_	81.92 d	9.95 c	1.39 d	3.45 a	82.23 d	9.08 c	1.27 d	3.61 a
**T**_**2**_	98.83 a	12.93 b	2.94 b	3.02 b	102.29 a	12.06 b	2.60 b	3.30 b
**T**_**3**_	86.92 c	12.99 b	2.01 c	2.89 c	89.75 c	12.12 b	1.74 c	3.00 c
**T**_**4**_	94.58 b	15.99 a	3.06 a	2.28 d	97.27 b	14.16 a	2.71 a	2.38 d
**LSD**	**1.61**	**0.33**	**0.09**	**0.03**	**1.61**	**0.31**	**0.09**	**0.03**
**V × T interactions**								
**V**_**1**_**T**_**1**_	91.00 f	11.55 fg	2.16 e	2.80 h	89.79 e	10.66 ef	2.03 de	2.93 g
**V**_**1**_**T**_**2**_	112.67 a	15.63 c	3.30 ab	1.93 m	115.79 a	14.85 b	3.00 a	2.14 k
**V**_**1**_**T**_**3**_	96.00 e	15.64 a	2.17 a	2.10 n	98.12 d	14.74 b	1.94 de	2.20 k
**V**_**1**_**T**_**4**_	106.00 b	17.52 a	3.38 a	1.34 n	108.21 b	16.22 a	2.95 ab	1.43 l
**V**_**2**_**T**_**1**_	84.00 g	10.48 h	1.25 g	3.12 ef	83.12 gh	9.70 g	1.14 g	3.27 e
**V**_**2**_**T**_**2**_	103.67 bc	13.21 d	3.16 bc	2.91 g	108.07 b	12.20 d	2.81 b	3.02 f
**V**_**2**_**T**_**3**_	89.00 f	14.01 d	2.23 e	2.62 i	92.21 e	12.89 c	1.89 e	2.77 h
**V**_**2**_**T**_**4**_	101.00 cd	16.34 b	3.28 ab	2.20 k	104.12 c	15.14 b	2.90 ab	2.31 j
**V**_**3**_**T**_**1**_	79.33 hi	9.49 i	1.11 gh	3.38 d	80.45 hi	8.58 h	1.02 gh	3.52 d
**V**_**3**_**T**_**2**_	98.00 de	11.83 f	2.99 c	3.07 f	101.11 cd	10.93 e	2.59 c	3.97c
**V**_**3**_**T**_**3**_	83.67 g	10.94 gh	1.87 f	2.90 g	86.55 f	10.64 ef	1.64 f	2.99 fg
**V**_**3**_**T**_**4**_	95.00 e	15.81 bc	3.14 bc	2.42 j	98.20 d	12.82 cd	2.91 ab	2.55 i
**V**_**4**_**T**_**1**_	73.33 j	8.26 j	1.03 h	4.50 a	75.54 j	7.36 i	0.91 h	4.74 a
**V**_**4**_**T**_**2**_	81.00 gh	11.04 gh	2.31 de	4.17 b	84.21 fg	10.26 fg	2.00 de	4.07 b
**V**_**4**_**T**_**3**_	79.00 hi	11.37 fg	1.76 f	3.94 c	82.12 gh	10.22 fg	1.50 f	4.05 b
**V**_**4**_**T**_**4**_	76.33 ij	14.27 d	2.42 d	3.16 e	78.54 ij	12.47 cd	2.08 d	3.24 e
**LSD**	**3.19**	**0.65**	**0.17**	**0.061**	**3.19**	**0.65**	**0.15**	**0.09**

DSI = disease severity index, V_1_ = Lasani-2008, V_2_ = Faisalabad-2008, V_3_ = Abdul Sattar-2002, V_4_ = Pasban-90, T_1_ = No fungicide application, T_2_ = Seed treatment, T_3_ = Foliar application at heading stage, T_4_ = Seed treatment plus foliar application at booting stage, any two means followed by same letter within a column are statistically non-significant, Units for plant height photosynthesis and chlorophyll are cm, μmoles CO_2_ m^−2^ s^−1^ and mg g^-1^, respectively

The addition of biological mulches (sugarcane and chickpea) and farmyard manure can reduce the incidence of KB. Planting cover crops with controlled irrigation during flowering and heading is helpful to manage the disease [28, 29]. A well-balanced irrigation and fertilization plan should be implemented during the cropping season to decrease KB risk. Wheat straw burning and polythene mulching after harvesting can increase soil temperature, which can destroy teliospores. Teliospores of KB can be disinfected by soil disinfection via cultural practices or fungicides [30, 31]. Application of some plants extracts like amaltas, neem and lantana under laboratory conditions have minimized the mobility of teliospores to 65%, but no successful results were observed under field conditions [9, 32].

### Disease severity index

Wheat cultivars, fungicide application timing and their interaction significantly altered disease severity index (DSI) during both years. The lowest DSI was noted for Lasani-08, whereas Pasban-90 had the highest DSI. Similarly, ST + FAH observed the lowest DSI, while NA had the highest DSI during both years (Table 4). Regarding cultivars × fungicide application timings’ interaction, Lasani-08 with ST + FAH had the lowest DSI, whereas Pasban-90 with NA recorded the highest DSI during both years (Table 4).

Pasban-90 is considered a susceptible cultivar to KB. Many researchers have used it as spreader in KB screening experiments. In earlier experiments, the highest disease incidence has been observed for Pasban-90 and AS-2002 [33]. Recently, KB is restricted to some developing countries. Different countries have already established well-developed quarantine rules for wheat imports to stop the mobility of KB. These countries are abiding strict measures as zero tolerance on import/export of wheat. Strict quarantine procedures have successfully managed KB in several European countries. One agreement was established in 1995 under world trade organization (WTO) to stop the spread of any pest/pathogen from origin country to other country. All the affiliated WTO states have adopted the phytosanitary practices as quarantine protocols to stop the entrance of harmful pathogens/pests. The WTO has recommended that every country should set strong identification and detection methods for harmful pathogens/pests at entry/exit points [9]. Many studies concluded that KB of wheat showed a significant reduction in disease severity after the application of fungicides [16]. Protective way (seed treatment and application on heading stage) is much effective against KB. The application of shelter (Mancozeb) and Dolomite (Metalaxyl+Mancozeb) showed a strong impact on teliospores of *T*. *indica* as protective spray on wheat under in vivo and in vitro conditions [34].

### Yield and related traits

Wheat cultivars, fungicide application timing and their interaction significantly altered yield and related traits during both years. The highest yield and related traits were recorded for Lasani-08, whereas Pasban-90 had the lowest values yield and poor yield-related traits during each study year. Similarly, ST + FAH observed the highest yield and related traits, while NA had the lowest yield and poor associated traits during both years (Table 4). Regarding cultivars × fungicide application timings’ interaction, Lasani-08 with ST + FAH had the highest yield and associated traits, whereas Pasban-90 with NA had the lowest values of these traits during both years (Table 5).

**Table 5:** The impact of fungicide application timings on yield and related traits of different wheat varieties having varying susceptibility levels to Karnal bunt disease.

	2016–17				2017–18			
Treatment	Spike length	Grains spike^-1^	1000-grain weight	Grain yield	Spike length	Grains spike^-1^	1000-grain weight	Grain yield
**Varieties (V)**								
**V**_**1**_	13.78 a	42.81 a	35.59 a	4259.08 a	13.84 a	40.21 a	33.96 a	3910.08 a
**V**_**2**_	12.57 b	38.78 b	32.74 b	3838.50 b	12.43 b	36.72 b	31.20 b	3470.75 b
**V**_**3**_	11.83 c	34.62 c	30.11 c	3752.83 d	8.55 d	32.40 c	27.55 c	3420.08 b
**V**_**4**_	10.96 d	30.38 d	27.49 d	3451.11 c	10.80 c	28.09 d	25.74 d	3138.11 c
**LSD 0.05**	**0.35**	**0.82**	**0.65**	**187.89**	**0.34**	**0.78**	**0.63**	**191.12**
**Application Timing (T)**								
**T**_**1**_	11.75 c	30.58 d	25.36 d	2328.50 c	11.25 b	26.07 d	23.98 d	2046.00 c
**T**_**2**_	13.39 a	41.10 a	35.05 b	4231.92 b	10.39 c	39.58 b	32.59 b	3829.42 b
**T**_**3**_	11.34 d	35.49 c	27.98 c	4059.03 b	11.33 b	33.98 c	26.62 c	3717.53 b
**T**_**4**_	12.66 b	39.43 b	37.53 a	4682.08 a	12.65 a	37.78 b	35.26 a	4346.08 b
**LSD 0.05**	**0.37**	**0.84**	**0.67**	**190.12**	**0.31**	**0.76**	**0.61**	**188.30**
**V × T interactions**								
**V**_**1**_**T**_**1**_	12.87 cd	36.03 e	29.23 fg	2752.67 g	12.37 de	30.44 g	28.03 fg	2454.67 f
**V**_**1**_**T**_**2**_	15.09 a	48.46 a	39.28 b	4404.00 bcd	15.42 a	47.25 a	37.38 a	3972.00 bcd
**V**_**1**_**T**_**3**_	12.99 c	41.43 c	32.01 e	4570.00 bc	13.31 c	39.53 d	30.78 e	4249.00 bc
**V**_**1**_**T**_**4**_	14.15 b	45.33 b	41.84 a	5309.67 a	14.27 b	43.63 b	39.64 a	4964.67 a
**V**_**2**_**T**_**1**_	11.67 ef	32.90 g	27.11 h	2404.67 gh	11.07 hi	28.01 h	26.09 h	2093.67 fg
**V**_**2**_**T**_**2**_	13.84 b	42.26 c	36.66 c	4314.33bcde	14.08 b	41.17 c	35.06 c	3879.33 cd
**V**_**2**_**T**_**3**_	11.86 ef	37.75 d	28.50 g	4030.00 de	11.78 efg	36.62 e	27.19 gh	3651.00 d
**V**_**2**_**T**_**4**_	12.91 c	42.20 c	38.67 b	4605.00 b	12.78 cd	41.08 cd	36.46 b	4259.00 b
**V**_**3**_**T**_**1**_	11.56 efg	28.07 h	24.61 i	2190.00 hi	11.13 ghi	25.04 I	23.01 I	1899.00 g
**V**_**3**_**T**_**2**_	12.88 cd	39.00 d	33.76 d	4209.33 cde	0.21 k	36.90 e	28.70 f	3811.33 d
**V**_**3**_**T**_**3**_	10.69 h	33.30 fg	27.07 h	4066.67 de	10.58 hi	31.63 fg	25.92 h	3745.67 d
**V**_**3**_**T**_**4**_	12.21 de	38.13 d	35.00 d	4545.33 bc	12.28 de	36.01 e	32.55 d	4224.33 bc
**V**_**4**_**T**_**1**_	10.90 gh	25.32 i	20.48 j	1966.67 i	10.45 i	20.80 j	18.78 j	1736.67 g
**V**_**4**_**T**_**2**_	11.74 ef	34.67 ef	30.51 f	4000.00 e	11.86 ef	33.02 f	29.21 f	3655.00 d
**V**_**4**_**T**_**3**_	9.81 I	29.47 h	24.36 I	3569.44 f	9.66 j	28.13 h	22.58 I	3224.44 e
**V**_**4**_**T**_**4**_	11.38 fgh	32.07 g	34.60 d	4268.33bcde	11.25 fgh	30.40 g	32.39 d	3936.33 bcd
**LSD 0.05**	**0.70**	**1.64**	**1.31**	**375.65**	**0.69**	**1.57**	**1.28**	**370.56**

V_1_ = Lasani-2008, V_2_ = Faisalabad-2008, V_3_ = Abdul Sattar-2002, V_4_ = Pasban-90, T_1_ = No fungicide application, T_2_ = Seed treatment, T_3_ = Foliar application at booting stage, T_4_ = Seed treatment plus foliar application at booting stage, any two means followed by same letter within a column are statistically non-significant, The units for spike length, 1000-grain weight and grain yield are cm, g and kg ha^-1^, respectively.

It is concluded from many studies that weight losses caused by KB vary from 2 to >50%. When infection ranges from 2–10%, it is considered that endosperm is partially damaged but if infection is >10% then whole endosperm/embryo is shattered. Grains having maximum infection display the substantial decline of seeds viability and result in weak seedlings. Infection level leads to eminence of wheat grains exaggeration. Wheat grains having infection <3% endure modest in terms of quality, while grains having infection >5% are unfit for eating [35–37].

The best physiological conditions for sprouting of *T*. *indica* teliospores are 20°C temperature and 15% or above soil water content [38, 39]. During the drying and freezing conditions, spores become dormant and resume their activity after the availability of favorable physiological conditions [9]. Many studies revealed the ideal moisture requirement for teliospores propagation on susceptible cultivars can be only provided by irrigation when average rainfall is minimal. It is observed that the incidence of KB is maximum in areas where moisture level is high. Teliospores have capability to survive in wet and dry soil conditions [40]. The soils where rice is grown (paddy soil) before the cultivation of wheat act as major source for teliospores’ survival [41]. The differences among experimental years can be owed to differences in climatic conditions faced by the plants and spores.

### Economic returns

Wheat cultivars, fungicide application timing and their interaction significantly altered economic returns during both years. The highest and the lowest net income and BCR were noted for Lasani-08 and Pasban-90, respectively during each study year. Similarly, ST + FAH observed the highest economic returns, while NA had the lowest net income and BCR during both years (Table 4). Regarding cultivars × fungicide application timings’ interaction, Lasani-08 with ST + FAH had the highest economic returns, whereas Pasban-90 with NA had the lowest economic returns during both years (Table 6).

**Table 6:** Economic analysis of different fungicide application timings on different wheat varieties having varying susceptibility levels to Karnal bunt disease.

	2016–17				2017–18			
Treatment	Total Cost	Gross income	Net income	BCR	Total Cost	Gross income	Net income	BCR
**Varieties (V)**								
**V**_**1**_	434.12	1140.83 a	706.71 a	2.63 a	448.02	1047.34 a	599.13 a	2.34 a
**V**_**2**_	434.12	1028.17 b	594.05 b	2.37 b	448.02	929.67 b	481.46 b	2.07 b
**V**_**3**_	434.12	1005.22 b	571.10 b	2.32 b	448.02	916.09 b	467.88 b	2.04 b
**V**_**4**_	434.12	924.40 c	490.28 c	2.13 c	448.02	840.57 c	392.36 c	1.88 c
**LSD 0.05**	**NS**	**50.32**	**50.32**	**0.11**	**NS**	**52.23**	**52.23**	**0.13**
**Application Timing (T)**								
**T**_**1**_	434.12	623.71 c	189.59 c	1.44 c	448.02	548.04 c	99.83 c	1.22 c
**T**_**2**_	434.12	1133.55 b	699.43 b	2.61 b	448.02	1025.74 b	577.53 b	2.29 b
**T**_**3**_	434.12	1087.24 b	653.12 b	2.50 b	448.02	995.77 b	547.56 b	2.22 b
**T**_**4**_	434.12	1254.13 a	820.01 a	2.89 a	448.02	1164.13 a	715.92 a	2.60 a
**LSD 0.05**	**NS**	**51.12**	**51.12**	**0.10**	**NS**	**51.12**	**51.12**	**0.12**
**V × T interactions**								
**V**_**1**_**T**_**1**_	434.12	737.32 g	303.20 g	1.70 g	448.02	657.50 f	209.29 f	1.47 f
**V**_**1**_**T**_**2**_	434.12	1179.64 bcd	745.52 bcd	2.72 bcd	448.02	1063.93 bcd	615.72 bcd	2.37 bcd
**V**_**1**_**T**_**3**_	434.12	1224.11 bc	789.99 bc	2.82 bc	448.02	1138.13 bc	689.92 bc	2.54 bc
**V**_**1**_**T**_**4**_	434.12	1422.23 a	988.11 a	3.28 a	448.02	1329.82 a	881.61 a	2.97 a
**V**_**2**_**T**_**1**_	434.12	644.11 gh	209.99 gh	1.48 gh	448.02	560.80 fg	112.59 fg	1.25 fg
**V**_**2**_**T**_**2**_	434.12	1155.63 bcde	721.51 bcde	2.66 bcde	448.02	1039.11 cd	590.90 cd	2.32 cd
**V**_**2**_**T**_**3**_	434.12	1079.46 de	645.34 de	2.49 de	448.02	977.95 d	529.74 d	2.18 d
**V**_**2**_**T**_**4**_	434.12	1233.48 b	799.36 b	2.84 b	448.02	1140.80 b	692.59 b	2.55 b
**V**_**3**_**T**_**1**_	434.12	586.61 hi	152.49 hi	1.35 hi	448.02	508.66 g	60.45 g	1.13 g
**V**_**3**_**T**_**2**_	434.12	1127.50 cde	693.38 cde	2.60 cde	448.02	1020.89 d	572.68 d	2.28 d
**V**_**3**_**T**_**3**_	434.12	1089.29 de	655.17 de	2.51 de	448.02	1003.30 d	555.09 d	2.24 d
**V**_**3**_**T**_**4**_	434.12	1217.50 bc	783.38 bc	2.80 bc	448.02	1131.52 bc	683.31 bc	2.52 bc
**V**_**4**_**T**_**1**_	434.12	526.79 i	92.67 i	1.21 i	448.02	465.18 g	16.97 g	1.04 g
**V**_**4**_**T**_**2**_	434.12	1071.43 e	637.31 e	2.47 e	448.02	979.02 d	530.81 d	2.18 d
**V**_**4**_**T**_**3**_	434.12	956.10 f	521.98 f	2.20 f	448.02	863.69 e	415.48 e	1.93 e
**V**_**4**_**T**_**4**_	434.12	1143.30 bcde	709.18bcde	2.63 bcde	448.02	1054.38 bcd	606.17 bcd	2.35 bcd
**LSD 0.05**	**NS**	**100.61**	**100.61**	**0.23**	**NS**	**101.45**	**101.45**	**0.26**

BCR = Benefit cost ratio, V_1_ = Lasani-2008, V_2_ = Faisalabad-2008, V_3_ = Abdul Sattar-2002, V_4_ = Pasban-90, T_1_ = No fungicide application, T_2_ = Seed treatment, T_3_ = Foliar application at booting stage, T_4_ = Seed treatment plus foliar application at booting stage, any two means followed by same letter within a column are statistically non-significant, The units for total cost, net income and gross income are $.

## Conclusion

Fungicide application timing and wheat cultivars significantly altered disease severity index, yield and economic returns of wheat. The cultivar with the highest tolerance level to the disease had the highest yield and economic returns and lowest disease severity index. Similarly, combination of fungicide application as seed treatment and foliar application at heading stage reduced disease severity index and improved yield and economic returns during both years. It is recommended that cultivars with higher tolerance level must be sown and fungicide should be applied as seed treatment and foliar application at heading to lower disease severity index and improve yield and economic returns of wheat.
